# Effects of Remimazolam Combined with Esketamine Anesthesia on Circulatory and Respiratory Function during Painless Gastroenteroscopy

**DOI:** 10.1155/2022/1079099

**Published:** 2022-10-12

**Authors:** Cheng Lu, Jun Ren, Xin Guo, Jiang Qian

**Affiliations:** ^1^Department of Surgical Anesthesia, China-Japan Friendship Hospital, Beijing, China; ^2^Department of Surgical Anesthesia, Xinjiang Corps Hospital, Xinjiang, China

## Abstract

**Objective:**

To investigate the effect of applying remimazolam combined with esketamine for anesthesia in painless gastroenteroscopy on patients' circulatory and respiratory function.

**Method:**

In this study, 106 patients who had undergone painless gastroenteroscopy in Xinjiang Production and Construction Corps (XPCC) Hospital between July 2021 and January 2022 were selected as study subjects, which were grouped according to the anesthetic drugs used in the surgery and divided into control group (*n* = 53 cases) and observation group (*n* = 53 cases), while those who were anesthetized with propofol + sufentanil during the operation were the control group and those who were anesthetized with remimazolam + esketamine were the observation group. To compare the induction time of anesthesia, patient awakening and recovery time of orientation, circulatory and respiratory function, intraoperative adverse effects, and postoperative complications in the two study groups.

**Results:**

There was no statistical difference in induction of anesthesia, patient awakening, and recovery time of orientation between the two groups (*P* > 0.05) and no statistical difference in postoperative complications (*P* > 0.05). The observation group had a better occurrence of local pain at the injection site, circulatory and respiratory function of patients after anesthesia, and intraoperative adverse reactions than the control group (*P* < 0.05).

**Conclusion:**

Remimazolam combined with esketamine anesthesia has the same advantages of rapid awakening compared with propofol anesthesia. Moreover, it has fewer side effects on patients' circulatory and respiratory functions with fewer adverse effects, as a suitable anesthetic method for painless gastroenteroscopy.

## 1. Introduction

Gastroscopy can directly observe the lesions in the patient's gastrointestinal (GI) tract, with high diagnostic and accuracy rates, which is a critical examination and treatment technique in gastroenterology. Painless gastroenteroscopy assisted with anesthesia can effectively reduce patient discomfort during the procedure, upgrade patient comfort, and facilitate gastroenterologists' operation, which has been widely used in clinical practice use [1, 2]. Currently, the commonly used anesthetic drugs in clinical practice include propofol, sufentanil, fentanyl, and dexmedetomidine. However, the effects of different drugs used in clinical practice vary, so it has been a focus of attention for anesthesiologists to choose a reasonable combination of anesthetic drugs for painless gastroenteroscopy to facilitate rapid recovery, improve intraoperative safety, and reduce the incidence of complications. Propofol is an intravenous anesthetic that is characterized by the rapid onset of action, short duration of action, and no accumulation in a short time, but it is prone to causing hypotension and respiratory depression which can occur at high doses [3]. Sufentanil is a commonly used opioid analgesic with strong analgesic efficacy which can reduce the amount of intraoperative sedation, but is prone to adverse effects such as respiratory depression and nausea [4]. Propofol combined with sufentanil is a commonly used method for painless GI anesthesia. Remimazolam is a novel, short-acting benzodiazepine with rapid onset of action and rapid recovery with inactive metabolites, which has lower side effects on circulatory and respiratory systems. Esketamine is a novel type of narcotic analgesic with strong analgesic efficacy and rapid onset of action, without significant effect on respiratory function [5]. This study aimed to investigate the effect and value of remimazolam combined with esketamine anesthesia on painless gastroenteroscopy by taking different anesthesia on the circulatory and respiratory function and intraoperative and postoperative safety of patients who had undergone painless gastroenteroscopy in our hospital, which is reported below.

## 2. Materials and Methods

### 2.1. Patients' General Information

In this study, 106 patients who had undergone painless gastroenteroscopy in XPCC Hospital between July 2021 and January 2022 were selected as study subjects. (1) The inclusion criteria include the following: those who met the indications for painless gastroenteroscopy; all were 20 to 75 years old and patients had no allergies or contraindications to any of the drugs associated with this study. (2) The exclusion criteria include the following: patients with potentially life-threatening circulatory and respiratory diseases which had not been adequately controlled; hepatic dysfunction (Child–Pugh class C or higher); coagulation disorders; cognitive dysfunction; and pregnant and lactating women. All study subjects were divided into a control group (*n* = 53 cases) and an observation group (*n* = 53 cases) using the random-number table method, and there was no statistical difference between the two groups compared with each other in terms of baseline information such as sex, age, BMI, and the American Society of Anesthesiology (ASA) classification (*P* > 0.05), see Table 1 for details.

### 2.2. Methods

Both the study groups were treated with painless gastroscopy and were fasted for 8 h and abstained from drinking for at least 2 h before the operation. The random-number table method was used to divide them into control and observation groups.

In the control group, propofol + sufentanil was used for anesthesia, and 0.1 *μ*g/kg sufentanil and 1.5–2 mg/kg propofol were pushed intravenously, while 0.3–0.4 mg/kg remimazolam and 1 mg/kg esketamine were pushed intravenously in the observation group. Gastroscopy starts when the patient is unconscious and the muscles are relaxed. When intraoperative somatic movement occurred, an additional 0.5 mg/kg of propofol was added each time in the control group and 0.1 mg/kg of remimazolam was added each time in the observation group to keep the patient unconscious and somatic movement during the operation until the end of the operation.

The consciousness criteria include the following [6]: patients with a modified Aldrete score ≥9 was scored as awake.

The SpO_2_ decline criteria include the following: patients with SpO_2_ ≤90% and are recoverable after implementation of the measures.

The respiratory depression criteria include the following: patients with SpO_2_ ≤90%, duration of decline >10 s, and ineffective after implementation of improvement measures.

The intraoperative hypotension criteria include the following: patients with the degree of systolic blood pressure decreases >20% or mean pressure value < 80 mmHg in the study subjects after anesthesia and during the progress of surgery.

The criteria for intraoperative bradycardia include the following: patients with heart rate ≤50 beats/min.

### 2.3. Observation Indexes

(1) The anesthesia induction time, recovery time, and directional recovery time were compared between the two groups. (2) The circulatory and respiratory functions of the two groups before and after anesthesia were compared. (3) The adverse reactions during the progress of examination/procedure were compared between the two groups. (4) The complications after examination/operation were compared between the two groups.

### 2.4. Statistical Analysis Methods

In this study, the data related to this study were statistically analyzed by using the statistical software SPSS 22.0, in which the count data were expressed as (number of cases (percentage)), that is, *n* (%), and the chi-square (*χ*^2^) test was performed for the count data between the two groups; the measurement data were expressed as (mean ± standard deviation), that is, (±*s*), and the *t*-test was performed for the measurement data between the two groups. The *t*-test was performed for the measurement data between the two groups; *P* < 0.05 indicates the difference between the two groups after the corresponding test for the data compared.

## 3. Results

### 3.1. Anesthesia Induction, Patient Awakening, and Orientation Recovery Time

In this study, statistical analysis of induction of anesthesia, patient awakening, and orientation recovery time in the two study groups showed no significant difference in induction of anesthesia, patient awakening, and orientation recovery time between the two anesthesia protocols, but both were more rapid (*P* > 0.05), see Table 2 for details.

### 3.2. The Circulatory and Respiratory Function of Study Subjects before and after Anesthesia

Comparing the circulatory and respiratory functions of the two groups before and after anesthesia, it was found that the average arterial pressure (map), heart rate (HR), respiratory rate (RR), and SpO_2_ levels of the two groups before anesthesia were not statistically significant (*P* > 0.05). The levels of the map, HR, RR, and SpO_2_ in 53 subjects in the observation group after anesthesia were higher than those in 53 subjects in the control group (*P* < 0.05), see Table 3 for details.

### 3.3. Occurrence of Adverse Reactions during the Examination

A total of 38 of the 106 study subjects in this study experienced adverse reactions during the progress of the examination, accounting for 35.85% (38/106) of the total study subjects, of which a total of 4 study subjects experienced hypotension during the progress of the examination, accounting for 3.77% (4/106) of the 106 study subjects; 7.55% of the study subjects experienced bradycardia (8/106); a total of 4 patients (3.77% (4/106) of the total study subjects) with decreased oxygen saturation; 8.49% (9/106) with respiratory depression; and 12.26% (13/106) with local pain at the injection site. A comparison of the occurrence of adverse events during examination/procedure progression between the two groups showed that the 53 study subjects in the observation group had lower occurrences of hypotension, bradycardia, decreased oxygen saturation, the occurrence of respiratory depression, transient local pain at the injection site, and total adverse events during examination/procedure progression than the 53 study subjects in the control group (*P* < 0.05), see Table 4 for details.

### 3.4. Complication Status after Examination/Operation

A total of 11 (10.38%) of the 106 study subjects selected for this study developed complications after the examination/surgery, of which a total of 4 (3.77%) developed nausea after the examination/surgery, 4.72% (5/106) developed vomiting, and 3 (2.83%) developed rigor and a comparison of the two groups of postexamination/surgery The occurrence of complications were compared between the two groups and found to be statistically insignificant (*P* > 0.05), see Table 5 for details.

## 4. Discussion

Esketamine is currently a relatively novel anesthetic drug with sedative and analgesic effects in clinical operations, which has the characteristics of rapid onset of action, strong anesthetic potency, less intraoperative drug dosage, shorter postoperative patient awakening time, and higher controllability than other anesthetic drugs, while its effect on the patient's circulatory and respiratory system function is lighter, often not inhibiting respiration and circulatory function excitation is lighter, but when we applied it alone in surgical therapeutic operations, it can postoperatively cause patients to nausea, vomiting, other GI system's adverse reactions, and myoclonic movements [6, 7]. Remimazolam is a benzodiazepine, which has the characteristics of rapid onset of action, rapid postoperative drug recovery, and lighter inhibition of circulatory and respiratory functions than other anesthetic drugs and can reduce neuronal excitability by acting on GABA receptors, causing a reduction in the body activity and sedation, but it can cause postoperative complications such as neurological and memory dysfunction in patients, without analgesic effect. Therefore, it is often used in combination with other analgesic anesthetic drugs [8, 9].

A total of 38 of the 106 study subjects in this study experienced adverse reactions during the progress of the examination, accounting for 35.85% (38/106) of the total study subjects, of which a total of 4 study subjects experienced hypotension during the progress of the examination, accounting for 3.77% (4/106) of the 106 study subjects; 7.55% of the study subjects experienced bradycardia (8/106); a total of 4 patients (3.77% (4/106) of the total study subjects) with decreased oxygen saturation; 8.49% (9/106) with respiratory depression; and 12.26% (13/106) with local pain at the injection site.

In this study, the induction of anesthesia, patient awakening, and recovery time of orientation were statistically analyzed in both the groups, and the results showed that the induction of anesthesia, patient awakening, and recovery time of orientation were rapid in both the groups, but there was no difference (*P* > 0.05); comparing the circulatory and respiratory functions before and after anesthesia in both the groups, it was found that the mean arterial pressure, heart rate, respiratory rate, and SpO_2_ levels were not statistically significant and were comparable (*P* > 0.05). The circulatory and respiratory functional status of all 53 study subjects in the observation group after anesthesia was superior to that of the 53 patients in the control group (*P* < 0.05), which was similar to the previous studies [10, 11]. Meanwhile, among the 106 study subjects in this study, a total of 25 study subjects had adverse reactions in blood pressure, heart rate, SpO_2_, respiration, and other vital signs during the progress of the examination/surgery, accounting for 35.85% (38/106) of the total study subjects, among which a total of 4 patients (3.77%) of the 35 study subjects who had adverse reactions had hypotension (4/106); 7.55% of the study subjects had bradycardia (8/106); a total of 4 patients (3.77% of the total study subjects) had decreased oxygen saturation; 8.49% (9/106) of the patients had respiratory depression; and 13 patients (12.26%) had transient local pain at the injection site. Among the abovementioned adverse events and total events, hypotension, bradycardia, decreased oxygen saturation, respiratory depression, local pain at the injection site, and the total incidence of adverse reactions were lower in the observation group (0.00%, 1.89%, 0.00%, 1.89%, 0.00%, and 3.77%) than in the control group (16.98%, 20.75%, 24.53%, 15.09%, 24.53%, and 77.36%) were lower (*P* < 0.05). A total of 11 (10.38%) of the 106 study subjects selected for this study had complications after the examination/surgery, including 4 (3.77%) patients who experienced nausea after the examination/surgery, 5 (4.72%) patients who experienced vomiting, and 3 (2.83%) patients who experienced rigor. The incidence of the abovementioned complications in the 53 study subjects in the observation group was 1.89% (1/53) for complicated nausea, 3.77% (2/53) for vomiting, 1.89% (1/53) for rigor, and 7.55% (4/53) for total postexamination/procedure complications; in the control group, the total incidence of nausea, vomiting, rigor, and postexamination/procedure complications were 5.66%, 5.66%, 3.77%, and 13.21%, respectively. It is consistent with the previous studies [11].

In conclusion, the use of remimazolam in combination with esketamine for painless gastroenteroscopy has the same advantages of rapid awakening time compared with propofol anesthesia, and it has fewer side effects on patients' circulatory and respiratory functions and fewer adverse effects, which can be a suitable anesthetic method in painless gastroenteroscopy.

## Figures and Tables

**Table 1:** Comparison of baseline information between the two groups (*n* (%), (false ± *s*)$\bar{x}$).

Groups		Observation groups (*n* = 53)	Control groups (*n* = 53)	*t/χ * ^2^	*P*
Sex (cases)	Male	29 (54.72)	31 (58.49)	0.154	0.695
	Female	24 (45.28)	22 (41.51)		

Age (y)		52.36 ± 6.45	51.32 ± 5.43	0.898	0.371
BMI (kg/m^2^)		23.88 ± 2.12	24.11 ± 2.52	0.508	0.612

ASA	Level I	23 (43.40)	25 (47.17)	0.152	0.696
	Level II	11 (20.75)	13 (24.53)	0.215	0.643
	Level III	19 (35.85)	15 (28.30)	0.693	0.405

**Table 2:** Comparison of anesthesia induction, patient awakening, and orientation recovery time in the two study groups (false ± *s*)$\bar{x}$.

Groups	Anesthesia induction time (s)	Patient awakening time (min)	Orientation recovery time (min)
The observation group (*n* = 53)	33.56 ± 7.61	11.12 ± 5.31	23.98 ± 6.22
The control group (*n* = 53)	36.52 ± 7.82	13.21 ± 5.62	26.32 ± 5.96
*t*	1.975	1.968	1.978
*P*	0.051	0.052	0.051

**Table 3:** Comparison of the circulatory and respiratory functions in the two study groups before and after anesthesia (false ± *s*)$\bar{x}$.

Time	Groups	MAP (mmHg)	Heart rate (beats/min)	Respiratory rate (times/min)	SpO_2_ (%)
Before anesthesia	The observation group (*n* = 53)	98.14 ± 4.61	81.54 ± 3.42	17.11 ± 4.02	99.42 ± 0.28
	The control group (*n* = 53)	97.49 ± 3.76	82.11 ± 4.51	16.38 ± 2.79	99.46 ± 0.33
	*t*	0.795	0.733	1.086	0.673
	*P*	0.428	0.465	0.280	0.503

After anesthesia	The observation group (*n* = 53)	94.77 ± 3.72	78.83 ± 3.76	15.21 ± 4.83	98.42 ± 0.26
	The control group (*n* = 53)	85.03 ± 4.72	62.11 ± 5.42	12.46 ± 3.21	95.88 ± 0.54
	*t*	11.799	18.453	3.452	30.853
	*P*	<0.001	<0.001	<0.001	<0.001

**Table 4:** Comparison of intraoperative adverse reactions in the two study groups (*n* (%) cases).

Groups	Low blood pressure	Bradycardia	Decreased oxygen saturation	Transient local pain at the injection site	Respiratory depression	Total incidence
The observation group (*n* = 53)	0 (0.00)	1 (1.89)	0 (0.00)	0 (0.00)	1 (1.89)	2 (3.77)
The control group (*n* = 53)	4 (7.55)	7 (13.21)	4 (7.55)	13 (24.53)	8 (15.09)	36 (67.92)
*χ * ^2^	4.157	4.867	4.157	14.817	5.950	47.421
*P*	0.041	0.027	0.041	<0.001	0.015	<0.001

**Table 5:** Comparison of the two study groups in terms of the occurrence of postexamination/procedure complications (*n* (%), cases).

Groups	Disgusting	Vomiting	Rigor	Total incidence
The observation group (*n* = 53)	1 (1.89)	2 (3.77)	1 (1.89)	4 (7.55)
The control group (*n* = 53)	3 (5.66)	3 (5.66)	2 (3.77)	7 (13.21)
*χ * ^2^	1.039	0.210	0.343	0.913
*P*	0.308	0.647	0.558	0.339

## Data Availability

All supporting experiment data are available from the corresponding author upon request.
